# Research on Camouflaged Human Target Detection Based on Deep Learning

**DOI:** 10.1155/2022/7703444

**Published:** 2022-10-12

**Authors:** Wei Zhang, Qikai Zhou, Ruizhi Li, Fu Niu

**Affiliations:** Academy of Systems Engineering of Academy of Military Science of Chinese PLA, Beijing 100166, China

## Abstract

In the task of camouflaged human target detection, the target is highly integrated with the complex environment background, which is difficult to identify and leads to false detection and missed detection. A detection algorithm MC-YOLOv5s is proposed for the characteristics of camouflaged targets. The algorithm takes YOLOv5s as the basic framework. First, a multispectral channel attention module is embedded in the backbone feature extraction network, which enhances the network's ability to extract camouflaged target features, weakens the attention to the surrounding background, and effectively improves the algorithm's antibackground interference. Second, the original upsampling operation is replaced by a lightweight general upsampling operator to achieve effective fusion of high-resolution low-level feature maps and low-resolution high-level feature maps. Finally, the K-means++ clustering method is used to optimize the anchor boxes of the dataset target, and the sizes of the generated priori boxes are allocated to each detection layer, which increases the matching degree between the priori boxes and the actual target boxes, and further improves the detection accuracy of the algorithm. The training and verification were carried out on the military camouflaged personnel dataset (MCPD), the precision (P), recall (R), and mean average precision (mAP) of the MC-YOLOv5s algorithm reached 97.4%, 86.1%, and 94%, respectively. Compared to the original YOLOv5s model, mean average precision (mAP) is increased by 3.7 percentage points. The improved algorithm has better detection effect, is more sensitive to camouflaged targets, and achieves accurate positioning and identification of camouflaged human targets. If the proposed MC-YOLOv5s is applied to personnel search and rescue in complex battlefields and natural disaster environments, it can greatly improve personnel search and rescue efficiency and life survival rate, and reduce the consumption of human and material resources in rescue.

## 1. Introduction

In recent years, target detection technology has made great achievements in all walks of life and has been widely used in military and civilian fields [1, 2]. At present, with the continuous development of high and new technologies such as artificial intelligence and big data, in the military field, modern warfare has developed from the previous mechanization to an unmanned, information-based, and intelligent mode, and various cutting-edge weapons and equipment in various countries in the world are gradually being developed. The development and improvement in the direction of technology and intelligence, especially the detection technology of military targets, has obviously become the key technology of battlefield situational awareness [3]. For intelligent weapons and equipment, the first problem to be solved is to make them have keen observation and identification capabilities. Therefore, in the complex and changeable battlefield environment, it is of great strategic significance for us to automatically and quickly identify potential enemy military targets.

In the civilian field, target detection algorithms have played an important role in the fields of autonomous driving, intelligent navigation, medical image recognition, and search and rescue [4, 5]. Especially when a natural disaster strikes unexpectedly, it may cause a large area of houses to collapse and cause casualties, so the top priority is to rescue the survivors in the rubble in time. At this time, rescue robots and search and rescue drones played a major role in emergency rescue. Rescue robots can quickly identify and locate survivors and carry out rescue work in complex and changeable disaster sites, especially in narrow spaces where fire rescue personnel, search and rescue dogs, or other rescue equipment tools are difficult to reach quickly. Compared with traditional remote sensing images and high-altitude aerial photography technology, search and rescue drones with target recognition and positioning functions are more efficient. In the future, more advanced and mature target detection technology will be applied to equipment such as search and rescue robots or search and rescue drones, which can greatly improve the search and rescue efficiency of personnel.

At present, the existing target detection algorithms are not outstanding in the above-mentioned target detection effect in the complex environment, especially the detection of camouflaged human targets in the complex environment, which is more difficult than the conventional detection task. In addition, military camouflage technology mainly changes the surface characteristics of the target through color, texture, and various patterns to achieve the effect of integrating into the surrounding complex environment to achieve the purpose of stealth, and some camouflage effects even reach the level that the human eye cannot recognize [6]. Not only that, the field environment where military targets are usually located is relatively complex, such as mountains, snow, deserts, and bushes, which may contain various military targets, all of which have brought enormous challenges to existing target detection algorithms.

After research and analysis, the difficulty of camouflaged human target detection mainly has the following two points: (1) the concealment of the target is very high, and the recognition degree is very low. Due to the complex diversity of its own dyes, patterns, and lines, the target is extremely integrated with the surrounding environment, and the discrimination is low; (2) overlapping occlusion is more common. Since the loss of target feature information is proportional to the degree of occlusion, overlapping occlusion will cause the algorithm network to lose part of the camouflage feature information during the feature extraction process, which in turn makes the training of the neural network more difficult. Therefore, if a convolutional neural algorithm with high accuracy and strong generalization ability can be developed, it will have important practical significance for the rapid search and positioning of targets in the field of intelligent combat and battlefield search and rescue.

Traditional military target detection algorithms are mainly identified by HOG [7], SVM [8], DPM [9], and other methods. However, the feature extraction ability of such algorithms is not enough, which leads to the loss of most of the target feature information, so the detection task of military targets in complex environments is more difficult, especially in the task of camouflaged target detection, which generally shows poor results. Since 2012, with the continuous upgrading of computers, the performance of many hardware devices has become better and better, and the target detection technology based on deep learning has also ushered in its rapid development period. Great progress has been made. At present, the military camouflage target detection algorithms for deep learning can be simply divided into two categories: one is the two-stage detection model (two stage), which uses the method of first dividing the target candidate area, then classifying and regressing, and representing the algorithm. There are R-CNN, Fast R-CNN, Faster R-CNN [10], etc.; the second is a single-stage detection model (one stage), which uses a network to directly classify and regress the target, and the representative algorithm has SSD [11], EfficientNet [12], RetinaNet [13], and YOLO series [14–17].

At present, many studies have applied target detection algorithms based on deep learning to precise guidance, battlefield search and rescue, and other military fields, and have achieved good detection results. According to Wang et al., [18] applying the Faster R-CNN algorithm to the tank armor target detection task in a complex background, compared with the traditional classic algorithm, effectively improved the target recognition rate. According to Yu and Lv [19], in response to the problem of not high detection accuracy of the traditional detection algorithm, it further improved the detection accuracy of military targets by introducing methods such as improving the ResNet50-D residual network and dual attention mechanism. Deng et al. [20] introduced an attention mechanism to imitating human vision on the basis of the RetinaNet algorithm and increased the detection accuracy of the camouflage target to 93.1%. The above studies have achieved good results for the detection tasks of military camouflage, but there is still room for improvement in the detection accuracy.

Based on this, this paper makes the following three improvements on the basis of the YOLOv5s algorithm framework for the characteristics that the camouflaged human target is highly similar to the surrounding environment: first, the multispectral channel attention module (MCA) is introduced in the backbone feature extraction network of YOLOv5s. The attention mechanism is added to make the algorithm network, which has the same keen observation ability as the human eye, so as to improve the network's full extraction of the information of the camouflaged human target, strengthen the algorithm's attention and antibackground interference ability, and further solve the problem that the original algorithm is insufficient to extract the features of the camouflaged human target; the second is to use the lightweight general upsampling operator CARAFE to replace the original upsampling operation to strengthen the effective fusion of high-resolution low-level feature maps and low-resolution high-level feature maps, so that the upsampling operation focuses on camouflage target area and the background area, which are ignored to achieve the content perception effect, so as to reduce the false detection rate of the original algorithm; the third is to use the K-means++ clustering algorithm to optimize the target a priori frame, and reclustering the dataset to generate the size of the new a priori frame is allocated to each detection layer, which increases the matching degree between the a priori frame and the actual target frame, and further enhances the network's ability to detect overlapping occluded targets. Through the above three improvements, this paper proposes a human target detection algorithm MCA-CARAFE-YOLOv5s (hereinafter referred to as “MC-YOLOv5s”) for camouflage characteristics, which effectively improves the algorithm's detection accuracy of camouflaged human targets in complex environments.

The scheme in this paper is applied to the complex and changeable battlefield environment. It can realize the recognition ability of various weapons and equipment similar to human eyes, automatically and quickly identify potential enemy military targets, and assist commanders in making battlefield decisions and achieve the goal of defeating the enemy. At the same time, when human-machine natural disasters and man-made disasters come, rescue robots and search and rescue drones using this technology can quickly search and rescue survivors trapped in the rubble, and rescue robots can quickly find and locate in complex environments. Survivors replace or assist manual rescue at the disaster site, especially in small spaces (such as holes less than 1 meter in diameter) that cannot be reached by humans, dogs, or other detection equipment, and the rescue safety factor is higher. It can automatically search and locate lost ships and personnel from a high altitude and a wide range, which greatly improves the efficiency of personnel search and rescue and the survival rate of life, and greatly reduces the consumption of manpower and material resources. In conclusion, this solution has important practical application value in both military and civilian fields.

## 2. The Detection Algorithm for Camouflaged Human Objects Based on Deep Learning

### 2.1. The Basic Principle of YOLOv5 Algorithm

The YOLOv5 algorithm is a detection algorithm with excellent detection speed and detection accuracy. The algorithm consists of four parts: the Input, the Backbone, the Neck and the Prediction. Its network structure is shown in Figure 1. The first is the input terminal, Input, the size of the input picture is generally 640 × 640. The second part is the backbone feature extraction network, Backbone, which is mainly composed of Focus, Conv, C3, Spatial Pyramid Pooling (SPP) [21], and other structures. The Focus structure is mainly the process of slicing and splicing feature maps in order to retain more feature information, and Conv is the basic convolution process, which mainly performs three operations such as 2-dimensional convolution, regularization, and activation on the input feature map. The C3 module consists of several Bottleneck structures. The third part is the feature fusion network Neck, which consists of Feature Pyramid Networks (FPN) [22] and Path Aggregation Networks (PANet) [23] structures. The combination of the two further improves the model's ability to target Feature attention. The fourth part is the detection layer Prediction. The three detection layers correspond to the detection and recognition of large-, medium-, and small-scale targets, respectively. The YOLOv5 algorithm model has four versions: *s*, *m*, *l,* and *x* according to the number of network layers. The change in the number of structural layers is mainly realized by changing the two parameters of depth multiple and width multiple. Among them, YOLOv5s has the least number of network layers, a simpler structure and the fastest speed.

### 2.2. A Camouflaged Human Target Detection Model Based on Improved YOLOv5

The YOLOv5 detection algorithm is one of the typical and excellent single-stage target detection algorithms. However, in the task of camouflage target detection under complex background, because the complex environment background in the picture usually occupies more, so in the process of extracting feature information, it is easy to generate redundant environment background information, which makes it difficult for the network to effectively extract the target feature information, and with the deepening of the network structure, the target feature information is seriously lost, resulting in poor target detection results. Therefore, this paper proposes a human target detection algorithm MC-YOLOv5s aiming at the characteristics of camouflaged targets, such as high concealment, low discrimination, and overlapping occlusion, which effectively improves the shortcomings of the original YOLOv5 algorithm and realizes the accurate identification and rapid positioning of camouflaged human targets in complex environments.

The network structure of the improved algorithm MC-YOLOv5s is shown in Figure 2. Input is the input terminal, and the size of the input picture is generally 640 × 640. Backbone is the backbone feature extraction network, which consists of modules such as Focus, Conv, C3, SPP, and multispectral channel attention module (MCA). The Focus structure is to slice and splice the input feature map, and add a value at every pixel point in the horizontal and vertical directions. More image information is preserved. Conv is the basic convolution unit of YOLOv5, which sequentially performs two-dimensional convolution, regularization, activation, and other operations on the input. C3 is composed of several Bottleneck modules. Bottleneck is a classic residual structure. After the input passes through two convolution layers, the Add operation is performed with the original value to complete the residual feature transfer without increasing the output depth. SPP is a spatial pyramid pooling layer. SPP performs three maximum pooling operations of different sizes on the input and contacts the output results to splicing the output results, so that the output depth of the network is the same as the input depth. The MCA module is one of the improved methods in this paper. In the improved algorithm, the MCA module is embedded into the backbone feature extraction network to improve the algorithm's antibackground interference ability, focusing on the original algorithm's ability to extract the features of camouflaged human targets.

The Neck part is mainly composed of feature pyramid network FPN and path aggregation network PANet. The FPN and PANet structures realize the fusion and complementation of high-level features and low-level features, so that the network can obtain more original image information and more accurate target recognition. The FPN structure transfers the category features of the high-level large objects to the lower layers, and the PANet structure transfers the location features of the low-level large objects and the category and location features of the small objects upward. Among them, the lightweight general upsampling operator CARAFE (Content-Aware ReAssembly of FEatures) is one of the improved methods in this paper. In the improved algorithm, the CARAFE module is used to replace the upsampling operation in the original algorithm, and the high-resolution low-level feature maps and low-level feature maps are strengthened. The fusion of high-resolution feature maps can avoid the loss of target feature information, thereby reducing the probability of false detection and missed detection.

The Prediction part is the detection structure of the improved algorithm. Since the input image size of the network in this paper is 640 × 640, and the downsampling is used 5 times in the improved algorithm, the final feature map size is 20 × 20, 40 × 40, 80 × 80, input it into the Detect module, which is used to identify large-, medium-, and small-scale targets, corresponding to 640 × 640, and the receptive field of each feature map is 640/20 = 32 × 32, 640/40 = 16 × 16, and 640/80 = 8 × 8 size.

#### 2.2.1. Multispectral Channel Attention Module

The traditional channel attention module mainly lies in setting the weight function of various channel importances. For example, the channel attention module (Squeeze and Excitation Network, SENet) [24] performs Global Average Pooling (GAP) on channels. The weight of each feature channel is automatically obtained by means of learning, and then, the features of the target area are strengthened and the background information irrelevant to the target is weakened according to the learned weight. If there is information loss, the GAP operation can only obtain general features. Although this selection is simple and efficient, GAP cannot fully obtain the rich semantic information of the target area, and it is easy to cause the problem of false detection and missed detection of overlapping occlusion targets.

The literature FcaNet [25] proves that GAP is a special form of discrete cosine transform (DCT), that is, the lowest frequency component, and only using GAP is equivalent to ignoring many other useful frequency components in the feature channel. Among them, the multispectral channel attention module (MCA) and other attentions have the same starting point, but the multispectral channel attention module not only retains the global average pool but also uses in addition to the global average pool. The frequency components can solve the problem of information loss caused by only focusing on a single frequency, make the network model to pay more attention to important features, and filter out redundant features. For this reason, in view of the problem that the military camouflaged human target is highly integrated with the surrounding environment background and has a low degree of discrimination, this study adds a multispectral channel attention module (MCA) to the YOLOv5s backbone feature extraction network to help the model effectively capture-rich feature information. More accurately, we identify and locate military camouflage personnel. The MCA module structure is shown in Figure 3.

The calculation of the general two-dimensional discrete cosine transform is shown in formula (1). Among them, *f*_*h*,*w*_^2 *d*^ is the spectrum of the two-dimensional DCT, and *x*_*i*,*j*_^2 *d*^ is the input; H and W represent the height and width of the input feature map, and the latter part is the DCT weight.

(1) $$\begin{array}{c} \begin{array}{c} f_{h,w}^{2\;d}=\overset{H-1}{\underset{i=0}{\sum }}\overset{W-1}{\underset{j=0}{\sum }}x_{i,j}^{2\;d}\cos\;\left(\frac{\pi h}{H}\left(i+\frac{1}{2}\right)\right)\cos\left(\frac{\pi w}{W}\left(j+\frac{1}{2}\right)\right),\\ s.t.\;h\in \left\{0,1,\cdots ,H-1\right\},w\in \left\{0,1,\cdots ,W-1\right\}. \end{array} \end{array}$$

Assuming that *h* and *w* in the 2-dimensional DCT are 0, formula (2) can be obtained. Among them, cos(0)=1, the left half is the lowest frequency component of the 2D DCT. Therefore, the following formula can prove that it is proportional to GAP.

(2) $$\begin{array}{c} \begin{array}{c} f_{0,0}^{2\;d}=\overset{H-1}{\underset{i=0}{\sum }}\overset{W-1}{\underset{j=0}{\sum }}x_{i,j}^{2\;d}\cos\;\left(\frac{0}{H}\left(i+\frac{1}{2}\right)\right)\cos\left(\frac{0}{W}\left(j+\frac{1}{2}\right)\right),\\ =\overset{H-1}{\underset{i=0}{\sum }}\overset{W-1}{\underset{j=0}{\sum }}x_{i,j}^{2\;d}=gap\left(x^{2\;d}\right)HW. \end{array} \end{array}$$

In order to simplify the operation and facilitate the description, *B* is used to represent the weight component of the 2D DCT, namely,

(3) $$\begin{array}{c} B_{h,w}^{i,j}=\cos\;\left(\frac{\pi h}{H}\left(i+\frac{1}{2}\right)\right)\cos\;\left(\frac{\pi w}{W}\left(j+\frac{1}{2}\right)\right)\text{.} \end{array}$$

Combined with the above formula, the inverse transform of the 2D DCT is rewritten into the following form:

(4) $$\begin{array}{c} \begin{array}{c} x_{i,j}^{2\;d}=\overset{H-1}{\underset{h=0}{\sum }}\overset{W-1}{\underset{w=0}{\sum }}f_{h,w}^{2\;d}\cos\;\left(\frac{\pi h}{H}\left(i+\frac{1}{2}\right)\right)\cos\left(\frac{\pi w}{W}\left(j+\frac{1}{2}\right)\right),\\ =f_{0,0}^{2\;d}B_{0,0}^{i,j}+f_{0,1}^{2\;d}B_{0,1}^{i,j}+\cdots +f_{H-1,W-1}^{2\;d}B_{H-1,W-1}^{i,j},\\ =gap\left(x^{2\;d}\right)HW\cdot B_{0,0}^{i,j}++f_{0,1}^{2\;d}B_{0,1}^{i,j}+\cdots +f_{H-1,W-1}^{2\;d}B_{H-1,W-1,}^{i,j}\\ s.t\;i\in \left\{0,1,\cdots ,H-1\right\},j\in \left\{0,1,\cdots ,W-1\right\}. \end{array} \end{array}$$

It can be seen from the above formula that the features of the input image can be divided into combinations of different frequency components, and the GAP operation is only one of the frequency components. To introduce more information, the multispectral channel attention module adopts 2D DCT to fuse multiple frequency components. The specific operation is to first divide the input feature map *X* into *n* parts according to the number of channels, *C*′ = *C*/*n*, where *n* must be divisible by the number of channels *C*. Then, each part has a two-dimensional DCT frequency component corresponding to it, and *F* represents the preprocessing result of the multispectral channel attention module, which can be expressed as follows:

(5) $$\begin{array}{c} \begin{array}{c} F^{i}=2DDCT^{u,v}\left(X^{i}\right)=\overset{H-1}{\underset{h=0}{\sum }}\overset{W-1}{\underset{w=0}{\sum }}X_{:h,w}^{i}B_{h,w}^{u,v}\\ s.t\;i\in \left\{0,1,\cdots ,n-1\right\}, \end{array} \end{array}$$

where *F*^*i*^ ∈ *R*^*C*′^is the preprocessed dimensional multispectral vector, and [*u*, *v*] is the frequency component index corresponding to *X*^*i*^. Then, the frequency components of different parts are combined, and the specific calculation is shown in

(6) $$\begin{array}{c} F=cat\left(\left[F^{0},F^{1},\cdots ,F^{n-1}\right]\right)\text{,} \end{array}$$

where cat represents the vector concatenation, and *F* ∈ *R*^*C*^ represents the multi-spectral vector obtained. Finally, the entire MCA attention module can be represented by *m*, and its specific calculation is expressed as formula (7), where sigmoid and *f*_*c*_ represent the activation function and the mapping function, respectively.

(7) $$\begin{array}{c} m=sigmoi\;d\left(f_{c}\left(F\right)\right)\text{.} \end{array}$$

Since the MCA module can incorporate frequency components containing different kinds of information into the attention processing, more feature information can be extracted. With the deepening of the number of neural network layers, the feature information of the target to be detected is gradually lost. In this paper, considering the impact of different frequency components in the multispectral channel attention on the performance of the YOLOv5s detection framework, the first *k* frequency components with better performance are selected for comparative experiments, and the value of *k* is 4, 8, 16, or 32.  Table 1 presents the ablation experiments of the parameters of the MCA module.

MAP in Table 1 represents the mean average precision. Two points can be found from the experimental data: first, the YOLOv5s model with multispectral channel attention (MCA) embedded in the Backbone part, and the detection performance is higher than the original YOLOv5s network model, which fully verifies the correctness of using multiple frequency components in channel attention. Second, when the frequency component in the MCA module is 16, the network can obtain the best detection effect. Therefore, the frequency components of the MCA module in the subsequent experiments in this paper are all taken as 16.

#### 2.2.2. Upsampling Algorithm Improvements

The upsampling operation is an important step in the multiscale feature fusion network to fuse high-resolution low-level feature maps and low-resolution high-level feature maps. Effective upsampling operations can bring better multiscale prediction. The upsampling operation in the original YOLOv5s model is the method of nearest neighbor upsampling, as shown in Figure 4. The nearest neighbor upsampling algorithm uses the spatial position of the pixel to determine the upsampling kernel, only considers the subpixel neighborhood, and does not make full use of the target feature information. It can be regarded as a kind of “uniform” upsampling, and the perception range is general. Are very small, the size of the receptive field is only 1 × 1 , so a lot of feature map information is lost, and the rich semantic features required for camouflage target detection cannot be well captured.

Therefore, this paper replaces the original upsampling operation by introducing a lightweight general upsampling operator (Content-Aware ReAssembly of FEatures, CARAFE) [26], in order to strengthen the high-resolution low-level feature maps and low-resolution high-level feature maps. Fusion is to avoid the loss of target feature information, thereby reducing the probability of false detection and missed detection, and improving the detection accuracy of the algorithm for camouflaged targets in complex environments. CARAFE is mainly divided into two modules: the Kernel prediction module and the content-aware reassembly module.

The network structure of CARAFE is shown in Figure 5.

Assuming *X* ∈ *R*^*C*×*H*×*W*^ is the input feature map, then the process of generating the target feature map *Y* ∈ *R*^*C*×*σH*×*σW*^ can be divided into the following steps: first, for the *k*_enco de r_ × *k*_enco de r_ neighborhood *N*(*X*_*l*_, *k*_enco de r_) of each position *l*=(*i*, *j*) in the input feature map, we use the Kernel prediction module to predict the recombination kernel *W*_*l*′_ of each *l*′, and the specific calculation is as shown in the following formula:

(8) $$\begin{array}{c} W_{l^{\prime }}=\varphi \left(N\left(X_{l,}k_{enco\;de\;r}\right)\right)\text{.} \end{array}$$

Then, the Kernel prediction module will use the 1 × 1 convolution to compress the number of channels of the input *X* from *C* to *C*_*m*_, and the channel reduction will not only cause no loss of feature information but also reduce the amount of network parameters and computation. The specific operation of the Content Encoder is to use *k*_enco de r_ × *k*_enco de r_ convolution to convert the number of channels from *C*_*m*_ to *C*_*up*_, *C*_*up*_=*σ*^2^ × *k*_*up*_^2^, and *σ* is the upsampling multiple. Using a larger *k*_enco de r_ will expand the receptive field to capture semantic information in a large range, but the network complexity increases with the increase of *k*_enco de r_. The default parameters selected in this paper are as follows: *σ*=2, *k*_enco de r_=3, and *k*_*up*_=5. The resulting feature map of *H* × *W* × *σ*^2^ × *k*_*up*_^2^ is then restructured into a feature map of *σH* × *σW* × *k*_*up*_^2^ and then normalized using the Softmax function for the channel values at each location.

Finally, the weighted summation is performed on each *k*_*up*_ × *k*_*up*_ square area *N*(*X*_*upl*_, *k*_*up*_) centered on *l* = (*i*, *j*) in the feature map *σH* × *σW* × *k*_*up*_^2^ after the expansion to obtain the feature of the position *l*′(*i*′, *j*′) of the new feature map. Then, we perform feature reorganization to obtain the output feature map, and the specific calculation is shown in the following formula, where *r* = ⌊*k*_*up*_/2⌋.

(9) $$\begin{array}{c} Y_{l^{\prime }}=\overset{r}{\underset{n=-r}{\sum }}\overset{r}{\underset{m=-r}{\sum }}W_{l^{\prime }\left(n,m\right)}\cdot X_{\left(i+n,j+m\right)}. \end{array}$$

#### 2.2.3. K-Means++ Algorithm to Optimize Anchor Box

In YOLOv5, the method of adaptive anchor box is used to calculate the anchor box matching the target of the dataset. The core principle is to cluster all the target real boxes in the COCO dataset through the K-means clustering algorithm and finally get 9 cluster centers: (10, 13), (16, 30), (33, 23), (30, 61), (62, 45), (59, 119), (116, 90), (156, 198), and (373, 326), and each 3 is assigned to feature maps of large, medium, and small scales. The military camouflage personnel dataset constructed in this paper is mainly based on human targets, of which the target height is greater than the width of the vast majority. Obviously, the above a priori frame is difficult to meet the actual situation of human target detection, so the size of the a priori frame needs to be resized.

The K-means algorithm is a simple and practical clustering algorithm, which is easy to implement and has a good clustering effect. All values in the dataset were clustered according to known K values. The resulting cluster center is used to represent the center of each class and is obtained by averaging all the values in that class. However, the K-means algorithm has the following shortcomings: first, the K value needs to be given in advance, but this value is very difficult to estimate; second, the initial clustering center is randomly selected, and different initial values may produce different clustering effects. Once the initial value is not chosen well, it is likely to cause the algorithm to fail to converge, and eventually, only a local optimal solution can be obtained. The K-means++ clustering algorithm improves K-means. This method sets the distance between the initial cluster center points farther, which further reduces the number of operations, speeds up the algorithm, and can obtain more accurate clustering.

To this end, this paper uses the K-means++ clustering algorithm to re-optimize all the target real boxes in the military camouflage personnel dataset to improve the matching degree between the prior frame and the actual human target frame, and further accelerate the convergence speed of the network model. We improve the detection effect of military camouflaged human targets. In this paper, the 9 priori boxes generated by the K-means++ clustering algorithm are equally divided into 3 different prediction layers, and the size of the newly generated a priori boxes are shown in Table 2.

## 3. Dataset and Evaluation Indicators

### 3.1. Dataset

This paper uses the military camouflaged personnel dataset (MCPD) for experiments. The dataset mainly uses more than 60 military camouflage videos on the Internet in complex field environments as the original material, and initially captures 10,000 high-definition images of camouflage human targets (size of 1280 × 720) through video frame capture. Camouflage patterns in many countries. The target detection technology based on deep learning mainly relies on three important factors: data, algorithm, and computing power, in which high-quality data are the premise for the algorithm to accurately identify the target. Due to the randomness in the video clipping process, it has a great impact on the overall quality of the images in the dataset. Therefore, in order to avoid the influence of the quality of the dataset on the algorithm itself, this paper considers many factors such as multidirectional, multi-angle and target size, attitude, and clarity to screen the dataset images layer by layer, and finally retains relatively high-quality military camouflage target image.

After strict screening, the military camouflage personnel dataset (MCPD) contains a total of 1000 high-definition images, each image contains 1 to 3 camouflaged human targets, and then uses the image labeling tool LabelImg to calibrate the human targets in each image one by one. There are two types of human target and environmental background. Several characteristics of the military camouflaged personnel dataset (MCPD) constructed in this paper: (1) the target has high concealment and low discrimination; (2) the target scales are different, including human targets of various scales such as large, medium, and small; (3) various target postures, including upright, half-squat, lying down, frontal, back, and sideways; (4) the environmental background is complex, including 6 kinds of wild environments such as jungle, rainforest, mountain, desert, snow, and urban ruins, and many factors such as season, weather, light, and occlusion are also considered. Some image samples in the MCPD dataset are shown in Figure 6.

### 3.2. Evaluation Indicators

This paper selects the following four indicators as the evaluation criteria of the model: precision (P), recall (R), mean average precision (mAP), model size (MB), and processing image frames per second number of FPS (frames per second). Model inference speed FPS (frame/s) is obtained by averaging the detection time of 200 images in the test set under the server Tesla P100 graphics card environment. Among them, the calculation formulas of P, R, and mAP are shown in (10)–(13). Among them, TP (true positive) refers to samples that were originally positive and were classified as positive; FP (false positive) refers to samples that were originally negative but classified as positive, and FN (false negative) refers to samples that were originally positive but are classified as negative class samples.

(10) $$\begin{array}{c} P=\frac{TP}{TP+FP}\text{,} \end{array}$$

(11) $$\begin{array}{c} R=\frac{TP}{TP+FN}\text{,} \end{array}$$

(12) $$\begin{array}{c} AP=\frac{1}{n}\overset{n}{\underset{i=1}{\sum }}Pi=\frac{1}{n}P_{1}+\frac{1}{n}P_{2}+\ldots +\frac{1}{n}P_{n}\text{,} \end{array}$$

(13) $$\begin{array}{c} mAP=\frac{1}{C}\overset{C}{\underset{k=1}{\sum }}AP_{k}\text{.} \end{array}$$

In the above formula, the definition of accuracy P is as follows: the proportion of samples that are actually positive and predicted to be positive to all predicted positive samples, P pays more attention to the situation of wrongly classifying negative samples as positive samples, and the definition of recall R is as follows: actually, it is the proportion of samples that are positive and predicted to be positive to all actual positive samples. R pays more attention to classifying positive samples as negative samples. The average precision (AP) refers to the average of all the accuracies (i.e., the area under the PR curve) obtained under all possible values of recall. Mean average precision (mAP) refers to the mean of AP for each category. In formula, C (10) represents the number of classes, and *k* represents one class.

## 4. Results and Discussion

### 4.1. Experimental Environment

The experiments in this paper are based on the official open source project of YOLOv5 (version 5.0) using the YOLOv5s model as the basic configuration, the computer operating system is Ubuntu 18.04, the *Python* version is 3.8, the deep learning framework is Pytorch1.8.0, and the CPU processor is Intel (R) Xeon(R) Gold 6130 (memory size is 31 GB). All experiments were performed on a Tesla P100 (15 GB video memory), and CUDA (compute unified device architecture) and cuDNN (CUDA deep neural network library) were used for accelerated training in the experiments to improve the computing power of the computer.

### 4.2. Network Training

Before training, the military camouflaged personnel dataset (MCPD) is randomly divided into training set, validation set, and test set with a ratio of 6 : 2:2. In order to fully train the improved network model and prevent the neural network from overfitting, a variety of data enhancement methods are used to expand the dataset during training, including color transformation, left-right flip, translation zoom, and mosaic.

The number of training times, Epochs, is set to 100, the batch size is set to 32, the size of the input image is 640 × 640, the initial learning rate is 0.0001, the learning rate momentum and the weight decay coefficient are set to 0.937 and 0.0005, respectively, and the optimization strategy is Adam (adaptive moment estimation) [27] optimizer. After outputting the prediction results, the nonmaximum suppression algorithm is used to screen the prediction boxes.

### 4.3. Experiment Verification and Result Analysis

In this paper, two groups of experiments are designed for verification, which are different improved partial ablation experiments and different algorithm model comparison experiments.

#### 4.3.1. Ablation Experiment

In order to test the detection effect of the improved algorithm, an ablation comparison experiment was carried out: the MCA module, the CARAFE module, and the K-means++ algorithm were introduced into the original YOLOv5s model, respectively. The comparison of the ablation results is shown in Table 1. Among them, “√” indicates that the corresponding improvement method is used in the network model, and “×” indicates that the corresponding improvement method is not used in the network model.

From the data in Table 3, it can be seen that the introduction of multispectral channel attention (MCA) in the backbone feature extraction network of YOLOv5s increases the model size by only 18.7 MB. The precision (P), recall (R), and mean average precision (mAP) is increased by 0.7%, 0.6%, and 2.6%, respectively, indicating that the MCA module can enhance the attention to the target area of interest in complex environments, and effectively improve the original YOLOv5 algorithm network without attention preference and and effectively improve the problem that the original YOLOv5 algorithm network has no attention preference which leads to the loss of camouflage target feature information. The lightweight general upsampling operator CARAFE is introduced to replace the original upsampling operation, so as to strengthen the fusion of high-resolution low-level feature maps and low-resolution high-level feature maps, effectively solve the problem of false detection and missed detection, and make mean average precision (mAP) of the algorithm is increased by 0.7%, which effectively improves the detection accuracy. On the basis of the above improvements, the K-means++ clustering algorithm is used to re-optimize all the a priori boxes of the dataset, so that the size of the a priori boxes is more suitable for the real box of the human target, and the experimental data in the table show that the anchor frame optimization improves the detection effect of the network model to a certain extent. Compared with the original algorithm, the combination of the three has greatly improved the evaluation indicators, which fully shows that in the detection task of camouflaged human targets, adding the multispectral channel attention module can effectively weaken the complex background information in the picture and improve the resistance of the network. Background interference ability and the introduction of a lightweight general upsampling operator CARAFE can further strengthen the full fusion of low-level and high-level feature maps, so as to achieve a good detection effect. In summary, the improved algorithm achieves accurate detection and recognition of camouflaged human targets in complex environments.

#### 4.3.2. Comparison of Different Algorithm Models

In order to further verify the detection effect of the improved method in this paper, the improved algorithm is compared with several mainstream object detection models: RetinaNet, YOLOX, YOLOv5s, YOLOv5m, and YOLOv5l. The dataset and platform configuration conditions used in the experiment are the same, and the performance comparison results are shown in Table 4. The bold font is the optimal value of the project.

From the data in Table 4, it can be seen that the model size of the improved algorithm is only 33.1 MB, which is 18.7 MB higher than the original YOLOv5s algorithm, and the detection speed FPS is reduced by 31.2. However, the detection accuracy of the improved model for military camouflage personnel is improved by 3.7%. Compared with the four excellent algorithms such as RetinaNet, YOLOX, YOLOv5m, and YOLOv5l, the MC-YOLOv5s algorithm model is more lightweight and is superior to the appeal algorithm in terms of detection accuracy and inference speed. Overall, the improved algorithm has the best detection performance for camouflaged human targets.

### 4.4. Test Results

Figure 7 shows the detection results of camouflage personnel under typical complex backgrounds by five algorithms, including MC-YOLOv5s, YOLOv5s, YOLOX, YOLOv5m, and YOLOv5l. From the detection results in the figure, it can be seen that the improved algorithm has higher detection accuracy, can effectively capture the feature information of camouflage human targets, and has better detection performance.

## 5. Conclusions

In this paper, in the task of camouflaged human target detection in complex battlefield environments, there are problems that the target and the complex environmental background are highly integrated, and the detection effect is poor due to low discrimination. A human target detection algorithm MC-YOLOv5s based on the characteristics of camouflage is proposed. The algorithm introduces the multispectral channel attention module (MCA) in the backbone part of the backbone feature extraction network in YOLOv5s, which improves the network's full extraction of the feature information of camouflaged human targets and strengthens the ability to resist background interference; second, the lightweight general upsampling operator CARAFE is used to replace the upsampling operation in the original algorithm, and the high-resolution low-level feature map is further strengthened and the fusion of low-resolution high-level feature maps, reducing the false detection rate of the original algorithm. Finally, the K-means++ method is used to cluster the actual boxes of all objects in the dataset images to obtain the sizes of the more matching prior boxes. The combination of the three effectively solves the problem that the original YOLOv5s algorithm is difficult to fully extract the characteristics of camouflaged personnel and effectively integrate the underlying and high-level feature maps. At the same time, it improves the matching degree between the prior frame and the actual target frame, and strengthens the detection ability of the detection network to camouflage human targets in complex environments. The experimental results show that the MC-YOLOv5s algorithm has excellent detection effect on the MCPD dataset, and has stronger generalization ability. Compared with the original YOLOv5s algorithm model, the precision (P), recall (R), and mean average precision (mAP) are increased by 3.3%, 2.8%, and 3.7%, respectively. Detecting camouflaged personnel images in complex and changeable battlefield environments is better than algorithms such as RetinaNet, YOLOX, YOLOv5m, and YOLOv5l and significantly improves the two difficult problems of camouflaged human target detection mentioned above. If the proposed MC-YOLOv5s is applied to personnel search and rescue in complex battlefields and natural disaster environments, the efficiency of personnel search and rescue and the survival rate of life can be greatly improved, and the consumption of manpower and material resources in the rescue process can also be greatly reduced.

## Figures and Tables

**Figure 1:** YOLOv5s detection framework.

**Figure 2:** Network structure of MC-YOLOv5s.

**Figure 3:** Multispectral channel attention module.

**Figure 4:** Nearest neighbor upsampling.

**Figure 5:** Network structure of CARAFE.

**Figure 6:** Military camouflage target sample.

**Figure 7:** Comparison of detection results of different models.

**Table 1:** Performance analysis of different frequency components in MCA module.

Number	Backbone	Frequency	mAP/%
1	Backbone		90.2
2	Backbone + MCA	4	90.7
3	Backbone + MCA	8	90.5
4	Backbone + MCA	16	92.9
5	Backbone + MCA	32	91.1

**Table 2:** The priori box sizes.

Prior box size	Feature map scale		
	Big	Middle	Small
Anchor box 1	(32, 95)	(62, 241)	(96, 273)
Anchor box 2	(42, 138)	(75, 207)	(75, 207)
Anchor box 3	(53, 181)	(76, 29)	(143, 414)

**Table 3:** Comparison of ablation experiment results.

Model	MCA	CARAFE	K-means++	P/%	R/%	mAP/%	Size/MB
YOLOv5s	×	×	×	94.1	83.3	90.3	14.4
YOLOv5s	√	×	×	94.8	83.9	92.9	32.8
YOLOv5s	×	√	×	88.4	87.6	92.4	14.6
YOLOv5s	×	×	√	92.5	85.7	90.8	14.4
YOLOv5s	√	√	×	92.3	88.5	93.6	33.1
YOLOv5s	√	√	√	97.4	86.1	94	33.1

**Table 4:** Detection performance of different models.

Module	mAP/%	FPS	Size/MB
RetinaNet	81.4	6.4	138
YOLOX	88.7	13.4	34.3
YOLOv5s	90.3	**125**	**14.4**
YOLOv5m	92.6	45.5	40.4
YOLOv5l	93.4	43.5	93.7
MC-YOLOv5s	**94**	93.8	33.1

## Data Availability

No data were used to support this study.
